# Cationic Amino Acid Transporters and *Salmonella* Typhimurium ArgT Collectively Regulate Arginine Availability towards Intracellular *Salmonella* Growth

**DOI:** 10.1371/journal.pone.0015466

**Published:** 2010-12-03

**Authors:** Priyanka Das, Amit Lahiri, Ayan Lahiri, Minakshi Sen, Namrata Iyer, Nisha Kapoor, Kithiganahalli Narayanaswamy Balaji, Dipshikha Chakravortty

**Affiliations:** Center for Infectious Disease Research and Biosafety Laboratories, Department of Microbiology and Cell Biology, Indian Institute of Science, Bangalore, India; University of Hyderabad, India

## Abstract

Cationic amino acid transporters (mCAT1 and mCAT2B) regulate the arginine availability in macrophages. How in the infected cell a pathogen can alter the arginine metabolism of the host remains to be understood. We reveal here a novel mechanism by which *Salmonella* exploit mCAT1 and mCAT2B to acquire host arginine towards its own intracellular growth within antigen presenting cells. We demonstrate that *Salmonella* infected bone marrow derived macrophages and dendritic cells show enhanced arginine uptake and increased expression of mCAT1 and mCAT2B. We show that the mCAT1 transporter is in close proximity to *Salmonella* containing vacuole (SCV) specifically by live intracellular *Salmonella* in order to access the macrophage cytosolic arginine pool. Further, Lysosome associated membrane protein 1, a marker of SCV, also was found to colocalize with mCAT1 in the *Salmonella* infected cell. The intra vacuolar *Salmonella* then acquire the host arginine via its own arginine transporter, ArgT for growth. The *argT* knockout strain was unable to acquire host arginine and was attenuated in growth in both macrophages and in mice model of infection. Together, these data reveal survival strategies by which virulent *Salmonella* adapt to the harsh conditions prevailing in the infected host cells.

## Introduction

*Salmonella* are gram negative facultative intracellular bacteria that can infect a wide range of animal hosts through contaminated food or water. Typhoidal strains such as *Salmonella enterica* serovars Typhi and Paratyphi infect humans causing a life threatening systemic illness called typhoid fever. On the other hand, non typhoidal strains like *Salmonella* Typhimurium and Enteritidis have a broader host range and in humans it can cause acute gastroenteritis [1]. *Salmonella* have the unique capability to survive and replicate within macrophages and this property is essential for its ability to cause systemic infection [2]. In order to overcome and survive in the hostile environment prevailing inside the macrophages, *Salmonella* has evolved strategies to escape the host innate and adaptive immune mechanisms. Nitric oxide (NO) and Reactive oxygen species are the central component of host innate immunity and effective antimicrobial agent against intracellular pathogens. However, the survival of *Salmonella* in the macrophages suggests that the pathogen has evolved mechanisms to avoid these host immune responses [3].

The activity of iNOS is dependent on the arginine availability. Therefore, the amount of arginine present in the host cell and the arginine acquiring capacity of the host and pathogen might play an important role in shaping the fate of any infection [4]. Arginine is an essential modulator of the host immune response [5], [6]. It has been shown that the uptake of arginine from extracellular milieu is required for the iNOS dependent NO production [7]. It has been long known that classical activation of murine macrophages leads to increased arginine transport [8]. Several mammalian arginine transport systems have been documented including systems y^+^, B^0+^, b^0+^ and y^+^L [9]. Transport at the basal level in non activated macrophages happens through the y^+^L system and in the activated macrophages it occurs via the y^+^ system. The cationic amino acid transporter family (CAT) belongs to the y^+^ system and includes four members CAT1 to 4 encoded by *Slc7A1* to -*4* genes. Arginine is transported by the first three members of the cationic amino acid transporter family [10]. CAT1 is ubiquitously expressed except in liver while CAT3 is expressed only in brain. CAT2 has two splice variants of which CAT2A is expressed in the liver and smooth muscle cells and CAT2B in the macrophages [8].

Interestingly, arginine uptake is necessary not only for the host macrophages but also for the infecting pathogen. Several pathogens are known to alter the arginine metabolism inside the host cells both from pathogenic and cellular point of view [11], [12]. For example, intracelluar *Listeria* upregulates expression of the *arpJ* gene which is an arginine permease once within host [13]. *Mycobacterium marinum* induces *argS* gene which codes for an arginyl tRNA synthetase [14]. *Giardia lamblia* inhibits NO production inside the host macrophages by consuming all the arginine by a highly efficient arginine transport system [15]. In case of *Salmonella*, the presence of an arginine transport system is well documented. Thus, it can be expected that in order to survive the stringent nutrient conditions prevailing in the host cells, *Salmonella* might as well transport and utilize the host arginine for better growth and survival.

Therefore, our interest has been to determine whether the intracellular *Salmonella* can acquire macrophage arginine for growth and thereby reduce the cytosolic arginine availability for NO production. The aim of the present work was to study the effect of *Salmonella* infection on the host arginine pool. We observed that that *Salmonella* can indeed access the cytosolic arginine pool of the macrophages and use it for their protein synthesis by employing both the host and its endogenous arginine transporters.

## Results

### *Salmonella* infection increases arginine uptake in the infected host cells

After activation by various stimuli macrophages are known to increase arginine uptake [11]. Arginine is a crucial amino acid that dictates the fate of many infections by regulating the iNOS mediated NO production. Therefore, we went ahead to determine the effect of *Salmonella* infection on the arginine transport capacity of APCs. We measured the transport activity of BMDMs from the BALB/c mice after 12 h of *Salmonella* infection. Fig. 1A shows that *Salmonella* infection led to a marked increase in the arginine uptake capacity of the BMDMs. To further substantiate our finding, we examined the total cell population from the liver and spleen of the control and infected BALB/c mice. As expected, both liver and spleen cells, from the infected mice showed 3-fold more arginine uptake compared to cells from uninfected control mice (Fig. 1B). We next checked the arginine uptake capacity of DCs isolated from BALB/c mice.

**Figure 1:** *Salmonella* upregulates the arginine transport in Bone Marrow Derived Macrophages (BMDM), in mice liver, spleen and from dendritic cells. (**A**) The BMDMs were infected with WT *Salmonella* at a MOI of 10 and the arginine uptake assay was performed at 12 h post infection, (**B**) A cohort of 5 mice was inoculated orally with 1×10^6^ CFU of the WT strain and dissected after 5 days post infection. Uninfected (UI) mice were treated with PBS. Liver and Spleen cells from either the infected or UI mice were subjected to the arginine uptake assay. Data represented is one of the three similar experiments. Statistical significance was defined as follows: **, *P*<0.01 (Student's *t* test).

### *Salmonella* infection increases cationic amino acid transporter mCAT1 and mCAT2B level in BMDMs

To identify the mechanism by which *Salmonella* infection led to an increased arginine uptake by BMDMs, the total RNA was isolated from *Salmonella* infected and uninfected BMDMs derived from BALB/c mice for the quantification of mCAT1 and mCAT2B mRNA. Basal expression of both mCAT1 and mCAT2B mRNA was observed in the uninfected BMDMs. However, *Salmonella* infection for 12 h led to a significant increase of both the mCAT1 (5-fold) and mCAT2B (3-fold) mRNA compared to the uninfected macrophages (Fig. 2A–B). Our results are consistent with the hypothesis that Salmonella infection increases arginine uptake by increasing the expression of these two transporters.

**Figure 2:** *Salmonella* infection in the Bone Marrow Derived Macrophages (BMDM) increases the expression of the murine cationic amino acid transporter 1 (mCAT1) and murine cationic amino acid transporter 2 (mCAT2B). (**A**) The BMDMs were infected with the WT *Salmonella* at an MOI of 10 and the levels of mCAT1, mCAT2B and *β-actin* mRNA was examined by Semi quantitative RT-PCR at 12 h post infection. (**B**) The mean fold increase in mCAT1and mCAT2B transcription after infection from three independent experiments after densitometric analysis and normalization with *β-actin* is plotted. The levels are compared from the infected to the uninfected macrophages from those experiments. Statistical significance was defined as follows: * *P*<0.05 (Student's *t* test).

### *Salmonella* arginine permease *argT* is essential for acquiring the host arginine

We hypothesized that *Salmonella* is using the host arginine for growth. Next, we went ahead to check how the pathogen acquires the host arginine. We hypothesized that specific arginine transporter in the bacterial membrane might transport the host arginine to the bacteria. To prove this point, we examined the role of the lysine-arginine-ornithine-binding periplasmic protein ArgT encoded by the *argT* gene (STM 2355). The other genes present in the same operon are *hisP* and *hisMQ* which encode the ATP-binding component and two integral membrane components, respectively, of both the lysine/arginine/ornithine ABC transporter and the histidine ABC transporter of *E. coli* [16]–[18]. Bioinformatics analysis against non-redundant protein databases revealed that several arginine permeases from both nonpathogenic and pathogenic bacteria shared significant homology with *Salmonella* ArgT (data not shown).

To check whether ArgT protein is expressed by intracellular *Salmonella* we made a knock in strain where 6 histidine were tagged to the C terminal of the chromosomal ArgT protein. We observed only one single band of 27 kDa belonging to the histidine tagged ArgT protein. As checked by western blotting the control *Salmonella* lysate does not give rise to any other histidine tagged protein of any size. The same strain was used to infect the BMDMs and after 12 h of infection, bacteria were purified and lysed. The protein was used to measure the amount of ArgT protein expressed by the intracellular *Salmonella*. The same bacteria grown in LB for 12 h were used as a control. By comparing the amount of RRF protein expressed in the intracellular *Salmonella* and LB grown *Salmonella* from the knock in strain we observed that the ArgT protein gets upregulated by around 2 to 3-fold upon infection (Fig. 3A–B). The WT strain has been used as a negative control to show that *Salmonella* does not have any histidine tagged protein in itself.

**Figure 3:** ArgT is expressed by intracellular *Salmonella*. (**A**) The expression of the His tagged ArgT protein in LB grown and from isolated ArgT:: His knock in bacteria from infected BMDM after running SDS PAGE is shown. The WT control bacteria do not have any His tagged protein in the same size. Ribosome Recycling Factor (RRF) probing was done to equalize the amount of bacterial protein loaded for the SDS PAGE (**B**) The mean fold increase of the ArgT protein level after infection for 12 h when compared to the LB grown bacteria from three independent experiments after densitometric analysis and normalization with Ribosome Recycling Factor (RRF) was plotted. Statistical significance was defined as follows: * *P*<0.05, (Student's *t* test).

To elucidate the function of *argT*, we made a single gene knock out in the WT *Salmonella* and confirmed the strain mutation various sets of primers. The strain was not growth defective in either LB or M9 minimal media (data not shown). The arginine uptake capacity of the WT and the Δ*argT Salmonella* strain were next checked *in vitro* using radioactive arginine. The data presented in Fig. 4A clearly demonstrates that the Δ*argT* bacteria are not able to uptake exogenous arginine like the WT strain. The complement strain (c-*argT)* behaves similar like the WT strain. To further understand the fate of the host derived arginine in *Salmonella in vivo*, we infected BMDMs from BALB/c mice with either the WT, Δ*argT* or the c-*argT* strains in arginine free DMEM. After infection for 25 min, ^14^C-arginine was added. After 12 h of infection we isolated intracellular bacteria from the infected cells and the bacteria were plated in antibiotic plate to enumerate the number of bacteria present for the different strains. After obtaining the CFU data, bacterial number was normalized for the different samples and duplicate wells were used for further experiments. Whole bacterial protein after normalizing was loaded in SDS page and phosphor imager scan was performed after 12 h of exposure. The protein profile of the WT strain contained significant amount of radiolabelled arginine indicating that the bacteria has used the host cytosolic arginine pool for its own translation. However, the Δ*argT* strain did not incorporate the host radiolabelled arginine (Fig. 4B, upper panel). The complemented argT strain showed a protein profile similar to the WT strain. The equal loading of the proteins were confirmed by doing western blotting for the ribosome recycling factor (RRF) protein of *Salmonella* (Fig. 4B, middle panel). Host protein contamination was ruled out by doing a western blot for β-Actin). Data presented in Fig. 4B, lower panel shows that host protein is effectively removed from the samples as only in the positive control of BMDM lysate has β-Actin band.

**Figure 4:** *Salmonella* utilize host derived arginine for protein synthesis. (**A**) Arginine uptake assay was performed with 10^8^ numbers of the WT, Δ*argT* and the *argT* complemented strain (c- *argT)* in the late stationery phase of growth. (**B**) **Upper panel**, The BMDMs maintained in arginine free DMEM were infected with either the WT, Δ*argT* or the *argT* complemented strain (c- *argT)*. After 25 min of infection, radiolabelled arginine was added to the cells. After 12 h of infection equal amounts of the isolated bacterial proteins from 10^9^ bacteria were loaded on SDS page. The gel was exposed in the cassette for 12 h and the incorporated radioactivity was assessed by the phosphor imager scan. **Middle panel**, Equal loading of the bacteria in all the samples was confirmed by performing anti- Ribosome Recycling Factor (RRF) western blotting. **Lower panel**, Cellular contamination in the samples were checked by doing β-Actin western blotting. In the positive control with BMDM lysate only the specific band for Actin was observed. Statistical significance was defined as follows: **, *P*<0.01, **, *P*<0.01 (Student's *t* test).

### ArgT is an essential virulence determinant

We suspected that the inability to utilize host cytosolic arginine might hamper the Δ*argT Salmonella* survival inside macrophages. In accordance to our hypothesis, in BMDMs the WT fold replication was 9-fold from 2 to 12 hour, whereas the Δ*argT* strain fold replication was only 3-fold. The *c-argT* strain grew equally like the WT strains (Fig. 5A). We next examined the role of *argT* in *Salmonella* survival *in vivo*. After infecting the BALB/c mice with either the WT strain or the Δ*argT* strain, we analyzed the bacterial load in the spleen and liver. After 5 days of infection, the bacterial load of the Δ*argT* strain was significantly less in the spleen and liver compared to the WT strain (Fig. 5B–C). The bacterial load of the c-*argT* strain was almost equal to the WT strain in the spleen. However, in liver, the c-*argT* strain did not exactly grow like the wild type strain but the virulence was reverted significantly from the knock out strain. Together, these data suggest that *argT* is an essential virulence determinant of *Salmonella*. The decreased bacterial burden of Δ*argT* strain *in vivo* might be due to the enhanced NO response of the macrophages in case of Δ*argT* infection and also due to the inability of the Δ*argT* strain to acquire host arginine pool for translation.

**Figure 5:** Δ*argT Salmonella* is attenuated for virulence and shows reduced bacterial proliferation *in vivo*. (**A**) Intracellular survival assay. BMDMs were infected at 10 MOI with the WT, Δ*argT* or the *argT* complemented strain (c- *argT)*. Infected macrophages were lysed at 2 and 16 h post infection and the bacterial loads were determined in triplicate. 1×10^6^ bacteria each of the WT or Δ*argT* or the argT complement strain (*c-argT*) strains were inoculated orally to a group of 6 male BALB/c mice. After 5^th^ day of infection, homogenized samples of (**B**) spleen, (**C**) liver of the infected mice were plated on antibiotic plates and the colonies were counted. Result presented is one of three independent experiments. Statistical significance was defined as follows: *, *P*<0.05, **, *P*<0.01 (Mann-Whitney *U* test).

Further, the nitrite response of the infected macrophages in case of the Δ*argT* infection was significantly higher compared to the wild type infected cells (Fig. 6A) indicating that the arginine available for NO synthesis in the Δ*argT* infected cells is more. In the BMDMs the argT strain is 3 fold attenuated when compared to the WT strain. To rule out if this increase in the NO response was dependent on the less number of bacteria in the Δ*argT* infected BMDMs, we performed the same experiment using a higher MOI of 30 for the Δ*argT* strain. In that condition also the cells infected with the Δ*argT* strain produced enhanced nitrite in the supernatant. To understand whether more arginine availability can enhance the macrophage NO response, we infected macrophages with wild type *Salmonella* at varying arginine concentration. Data presented in Fig. 6B indicates that increasing the arginine concentration in the culture medium from 0.5 to 1 mM indeed enhanced the NO response of the WT infected macrophage cells. However, further increase of L-arginine form 1 mM to 2 mM had no effect on the nitrite production. Thus, the increased NO response of the Δ*argT Salmonella* infected macrophages may be due to more arginine availability to iNOS for NO synthesis.

**Figure 6:** The Δ*argT* strain infection in the BMDMs gives rise to high NO response. (**A**) BMDMs were infected at 10 MOI with the WT, Δ*argT* or the *argT* complemented strain (c- *argT*) and also with 30 MOI of the Δ*argT* strain and the *argT* complemented strain (c- *argT*) strain. Production of nitrite was determined in the culture supernatants of the infected BMDMs by Griess reaction after 12 h of infection. (**B**) BMDMs were maintained in 0.5, 1.0, 1.5 or 2.0 mM concentration of L-arginine and infected with the WT *Salmonella* for 12 h. Production of nitrite was determined in the culture supernatants by Griess reaction. Values are expressed as mean ±SD of one of three independent experiments performed in triplicate. Statistical significance was defined as follows: * *P*<0.05 (Student's *t* test).

### The mechanism of cytosolic arginine uptake by intracellular *Salmonella*

We next examined the mechanism by which intracellular *Salmonella* accesses the host cytosolic arginine pool. We checked for the colocalization of mCAT1 to intracellular *Salmonella* in BMDMs by confocal microscopy. We observed that the host mCAT1 which is exclusively expressed in the cell membrane in uninfected macrophages is preferentially recruited to the intracellular *Salmonella* in the infected BMDMs. We went ahead to check mCAT1 recruitment to intracellular *Salmonella* at different time points post infection. For this purpose, we infected macrophages with WT-GFP *Salmonella* for different time intervals (Fig. 7A, 8A) and observed that mCAT1 localization to the SCV starts after 3–4 h of infection. We also immuno-stained the infected cell for LAMP1, which is a marker of SCV, to conclusively demonstrate the localization pattern of the host CAT transporters. We observed significant amount of co localization of the WT viable *Salmonella* (green) and mCAT1 protein (red) after 4 h (Fig. 7C) and 12 h (Fig. 8C) of infection generating yellow colour. The LAMP1 protein (blue) also significantly colocalizes with bacteria (green) at both the time points generating cyan colour (Fig. 7B, 8B) indicating the presence of LAMP1 in the SCV. At both the time points 80–90% of the bacteria had cyan colour. Our data indicates that the mCAT protein is also recruited to the LAMP1 containing vacuole giving rise to magenta (data not shown) colour in the infected cell. The colocalization co efficiency of the total blue (LAMP1) with red (mCAT1) that has given rise to magenta colour is around 26% at 4 h of infection. This colocalization increases to 57% after 12 h of infection clearly pointing to the fact that *Salmonella* continuously recruit the mCAT1 protein to SCV. Similarly, after infection for 12 h, the amount of mCAT1 and bacterial colocalization increases than that of 4 h of infection clearly indicating the recruitment to be an active one. In multiple fields the amount of bacteria colocalized to the mCAT1 protein was calculated. This was done by dividing the number of bacteria having yellow spots to the total number of bacteria from various field and multiple experiments. 4 h of *Salmonella* infection in BMDMs allowed 35% of the total *Salmonella* to acquire mCAT1. 12 h of infection allowed almost 75% of the bacteria out of the total intracellular bacteria to recruit mCAT1 (Fig. 8E). Three kinds of colocalization were observed namely spot colocalization, partial colocalization or the full bacteria colocalization with the mCAT1 protein (Fig. 7C, 8C insets). LAMP1 and mCAT1 colocalization in the GFP *Salmonella* indicates that the host arginine transporters are present in very close viscinity of the SCV. This gives rise to the same bacteria having both LAMP and mCAT1 immuno-staining and white colour if all three are in the same region. Enlarged bacteria are shown in the insets (Fig. 7D, 8D). This experiment clearly suggests that host arginine transporters are recruited by intracellular *Salmonella* to their vacuole.

**Figure 7:** Intracellular *Salmonella* starts colocalizing with host mCAT1 in the BMDMs at early time point of infection. BMDMs were infected with WT *Salmonella* for 4 h. The sites of colocalizations were detected by immunostaining with an anti-mCAT1 antibody and a Cy5-conjugated secondary antibody and with an anti-LAMP1 antibody and a Cy3-conjugated secondary antibody. Cy3 staining was pseudo-coloured as blue. Samples were analyzed by confocal laser-scanning microscopy and representative images for the localization of the BCG-GFP (green) and the mCAT1 (red) and the LAMP1 (blue) are shown. (**A**) Representative image for the localization of the WT-GFP (green) in grey scale image. (**B**) Image for the localization of the WT-GFP (green) and LAMP1 (blue). The colocalization gives rise to cyan colour. Inset: enlarged image of the bacteria containing vacuole. (**C**) Image for the localization of the CAT1 (red) and WT-GFP (green). The colocalization gives rise to yellow colour. Inset: enlarged image of the bacteria containing vacuole. (**D**) Image for the localization of the CAT1 (red) and WT-GFP (green) and LAMP1 (blue). LAMP1 and mCAT1 colocalization in the GFP *Salmonella* gives rise to the same bacteria having both LAMP and mCAT1 immuno-staining, enlarged bacteria are shown in the insets.

**Figure 8 pone-0015466-g008:** Intracellular *Salmonella* colocalizes with the host mCAT1 in the BMDMs at late time point of infection. BMDMs were infected with WT *Salmonella* for 12 h and the staining was done as described earlier. (**A**) Representative image for the localization of the WT-GFP (green) in grey scale image. (**B**) Image for the localization of the WT-GFP (green) and LAMP1 (blue). The colocalization gives rise to cyan colour. Inset: enlarged image of the bacteria containing vacuole. (**C**) Image for the localization of the CAT1 (red) and WT-GFP (green). The colocalization gives rise to yellow colour. Inset: enlarged image of the bacteria containing vacuole. (**D**) Image for the localization of the CAT1 (red) and WT-GFP (green) and LAMP1 (blue). This gives rise to the same bacteria having both the LAMP and mCAT1 immuno-staining, enlarged bacteria are shown in the insets. The colocalization of the three colours gives rise to white colour. (**E**) The percent colocalization of WT *Salmonella* with mCAT1 at 4 (white bar) and 12 h (black bar) post infection. The colocalization (%) of WT-GFP *Salmonella* with mCAT1 is plotted after counting from 50 fields in three independent experiments. Out of total bacteria the number of yellow bacteria was counted in those fields and colocalization (%) was plotted. The amount of LAMP1 colocalized to the mCAT1 protein is also shown. For this purpose, the colocalization efficiency of Blue that colocalized with Red and gave rise to magenta colour was counted. Statistical significance was tested by comparing the 4 h values with that of the 12 h values an defined as follows:* *P*<0.05 (Student's *t* test).

In order to better understand whether this mechanism is utilized by other intracellular bacteria, we checked for mCAT1 colocalization to intracellular *Mycobacterium bovis* BCG. Interestingly, in the *M. bovis* BCG infected BMDMs also it was observed that mCAT1 significantly colocalizes to the intracellular BCG (Fig. 9A). In contrast, no signs of colocalization were noted for the heat killed dead *Salmonella* in BMDMs after 12 h of infection (Fig. 9B) clearly indicating that the recruitment of mCAT1 is a survival strategy of the live and virulent *Salmonella* and is independent of *Salmonella* LPS. BMDMs infected with non-pathogenic *E.coli* showed significantly less amount of colocalization with mCAT1 suggesting this recruitment to be a virulence strategy of the pathogenic bacteria (Fig. 9C). GFP latex beads also showed drastically reduced colocalization pattern (Fig. 9D). In the case of *Mycobacteria* infected cells 70% bacteria out of total bacteria counted in many fields colocalized with mCAT1 protein, whereas the heat killed *Salmonella*, *E.coli* or the bead containing cells had only 10–20% of the total number of bacteria or the bead colocalized to the mCAT1 protein (Fig. 9E).

**Figure 9:** mCAT1 distribution pattern in the BMDMs after infection with various other pathogens or conditions. (**A**) Intracellular *M. bovis* BCG (GFP) colocalizes with the host mCAT1 protein in BMDM after 12 h of infection. The sites of colocalizations were detected by immunostaining with an anti-mCAT1 antibody and a Cy5-conjugated secondary antibody. Samples were analyzed by confocal laser-scanning microscopy and representative images for the localization of the BCG-GFP (green) and the mCAT1 (red) are shown. Inset: enlarged image of the bacteria containing region. (**B**) Heat killed *Salmonella* (GFP) after 12 h of infection in BMDM is shown in green and mCAT1 shown in red. Staining was done as described earlier. (**C**) BMDMS were infected with the dh5a *E.coli* strain (GFP) at a MOI of 10 for 12 h and staining was done as described earlier. (**D**) BMDMs were allowed to phagocytose inert latex beads (GFP, Ratio of 1∶25) and fixed after 12 h post phagocytosis. Staining was done as described earlier. (**E**) The percent colocalization of BCG, Heat killed *Salmonella* (HK), *E.coli* or GFP beads (Beads) with mCAT1 are plotted after counting from 50 fields in three independent experiments. Out of total bacteria/bead the total number of yellow bacteria/beads was counted in those fields and colocalization (%) was plotted and the significance was tested after comparing any group with the GFP-Bead's colocalization values. Statistical significance was defined as follows:* *P*<0.05 (Student's *t* test).

## Discussion

Arginine is a crucial regulator of the innate immune response of the host [5], [6]. There are two major transporters of arginine in the mammalian cells [8] and it has been reported that of these mCAT2B is required for sustained NO production in the macrophages [19]. Published reports suggest that the LPS and IFNγ treatment [20] or different pathogenic interference [21] can increase the expression of mCAT1 and mCAT2B arginine transporters. Previous studies have demonstrated that the survival of *M. bovis* [22], *Taxoplasma* [23],*Trypanosoma* [24] and *Leishmania* [25], [26] inside the macrophages depend on their ability to interfere with the arginine metabolic pathway of the host. We hypothesized that intracellular *Salmonella* might utilize the host cytosolic arginine in order to save on its own energy expenditure. Further, we were mainly interested in arginine transport as this amino acid is the only substrate for host NO production, which in turn can kill pathogenic *Salmonella*. We showed that after 12 h of *Salmonella* infection in the BMDMs, the mCAT1 and mCAT2B mRNA as well as arginine uptake was significantly up regulated compared to the uninfected cells. The liver and spleen cells of *Salmonella* infected mice also showed an enhanced arginine uptake. We further observed that even in the dendritic cells *Salmonella* infection led to an increased arginine uptake.

We hypothesized that the intracellular *Salmonella* can access the host cytosolic arginine pool by recruiting the arginine transporter from the cell membrane to SCV membrane. Our confocal data clearly demonstrated that intracellular *Salmonella* recruits the host arginine transporter mCAT1 to the bacteria containing vacuole. When in the infected cells we immuno stained for mCAT1 and LAMP1. Immediately following invasion, individual *Salmonella* are found within discrete vacuoles characterized by the transient presence of early endocytic markers on the membrane [27]. By 5–10 min post invasion, these proteins are replaced by lysosome-associated membrane proteins (LAMPs), which accumulate further over many hours [28]. LAMP1 is a known marker of SCV [29] and our data showed that more than 90% of the total bacteria were colocalized with LAMP1. We also observed that the mCAT1 protein gets recruited to the SCV. 4 h after infection around 35% of the total bacteria are colocalized with mCAT1. At late time point of infection this percentage increases to 75% indicating this recruitment to be an active process. We also observed that the mCAT1 protein and the LAMP1 are in close proximity in the infected cell and the colocalization increases actively with infection. On one hand, the colocalization of mCAT1 with bacteria and on the other, the colocalization of mCAT1 with previously known SCV marker LAMP1 clearly indicates the fact that host arginine transporters are recruited to SCV. This gives rise to the same bacteria having both LAMP and mCAT1 immuno-staining. Interestingly, this recruitment of mCAT1 is not shown by heat killed *Salmonella* or non-pathogenic *E.coli* or latex beads. Thus, the altered trafficking of mCAT1 appears to be an active process mediated by live pathogenic bacteria and is independent of LPS. Data presented in Fig. 7–[Fig pone-0015466-g008] 9 clearly shows that in case of Bead, *E.coli* or Heat-killed bacteria infected BMDMs; host mCAT1 is localized to the membrane. However, in case of *Salmonella* infection there is a clear redistribution. In the infected cell, the membrane as well as the SCV contains significant amount of the host arginine transporter. The fact that similar phenotype was observed with intracellular *M. bovis* BCG increases the importance of this novel discovery. Since, previous studies have depicted that in case of BCG infection there is a clear increase in the arginine uptake of host and in the expression level of the host arginine transporters. Further, the role of a *M. bovis* BCG gene, *gabP* is well established in the uptake of host arginine by intracellular BCG [12]. Our study provides the first evidence that the host arginine transporter mCAT1 is actually recruited to intracellular BCG. We wanted to examine whether CAT2B is also recruited to SCV after *Salmonella* infection. However, due to unavailability of commercial antibody we could not perform the confocal studies. In order to overcome this problem, we constructed cDNA-GFP construct of the murine CAT2B gene and transfected in the BMDMs. We observed colocalization of the GFP protein with SCV after *Salmonella* infection indicating that CAT2B also plays a major role to channelize host arginine to bacteria (data not shown). However, due to fusion of the GFP protein to the membrane transporter CAT2B there was a problem in the membrane spanning property of the protein. We observed diffused expression pattern of the CAT2B:: GFP construct throughout the cell.

We further hypothesized that the intra vacuolar *Salmonella* employs its endogenous arginine transporter to transport arginine from the host cytosol to inside the SCV. In accordance with our hypothesis, we observed a very critical role of an arginine periplasmic binding protein, ArgT, in *Salmonella* pathogenesis. The ArgT protein was found to be upregulated upon infection in the BMDMs indicating its role in the intracellular survival of *Salmonella.* As observed earlier [30], we also found out that this protein is not highly upregulated upon infection as this gene has role for in vitro survival as well. The *argT* knockout *Salmonella* was significantly attenuated in BMDMs and in the mice model of infection suggesting the fact that ArgT is the main arginine transporter in *Salmonella* required to acquire the host arginine and is an important virulence marker. In the Δ*argT* infection in BMDMs, the host NO response was significantly higher compared to wild type *Salmonella* suggesting this transport is also a mechanism to reduce host NO production by sequestering arginine away from the iNOS pathway. To further verify this point, we supplemented increasing amount of L-arginine during infection of the BMDMs with WT *Salmonella*. As observed earlier [31], the NO production from the infected macrophages enhanced significantly after altering the L-arginine concentration from 0.5 to 1 mM. Further increase of the L-arginine concentration had no added effect on the NO production as the substrate concentration for iNOS might have reached the saturation limit. To examine the fate of host arginine in *Salmonella* pathogenesis we tracked the incorporation of host radiolabelled arginine in wild type and Δ*argT Salmonella*. Phosphor imager showed that wild type *Salmonella* utilized host radiolabelled arginine for its own protein synthesis. The Δ*argT Salmonella* was not able to utilize the host arginine for its translation. To our knowledge, this study demonstrated for the first time that intracellular *Salmonella* utilizes the host arginine for survival in the antigen presenting cells like BMDMs and DCs. Interestingly, this uptake of host arginine by intracellular *Salmonella* can be used for specific delivery of arginine tagged antibiotics to the pathogen enabling better killing. Undoubtedly, host cell increases its arginine uptake in response to LPS during *Salmonella* infection to increase the iNOS activity and NO production to control the pathogen. However, *Salmonella* subverts this host defense mechanism and utilizes this extra arginine for its own translation.

In conclusion, the increase in host arginine transporters in response to *Salmonella* infection is an innate immune mechanism originally intended to increase the host NO production. However, our data provides evidence that this innate immune response intended to control the infection is being exploited by the pathogen for its own translation. Briefly, *Salmonella* infection increases the arginine transporters and the transporters get localized to the SCV. All these mechanisms lead to the uptake of arginine by the bacteria. Thus, *Salmonella* upregulates the host arginine transporters and utilizes the extra arginine. In this manner, *Salmonella* quenches arginine away from the iNOS pathway. In addition, the bacteria acquire arginine for their own protein synthesis at no extra cost. The energy advantage of this pathogenic strategy suggests that there may be possibly other amino acid transporters which get upregulated as well. However, we have not discussed them here as they are beyond the scope of our findings. Better understanding of the nutrient requirement of the pathogen will provide important clues towards further understanding this question. The elucidation of *Salmonella* effectors involved in the altered trafficking of the host arginine transporters awaits further studies. Our data indicates that the arginine tagged antibiotic might facilitate specific and targeted delivery of any antibiotic to intracellular *Salmonella* and *Mycobacteria* enabling better killing. In the infected cell, the arginine tagged antibiotic can reach the pathogen containing vacuole by means of the relocalized host arginine transporters and can prove to be very effective.

## Materials and Methods

### Ethics Statement

All the work with animals has been done with Institution approved ethics protocol. The ethics number being CAF/ETHICS/189/2010.

### Bacterial strains, media and growth conditions

The nalidixic acid resistant wild type (WT) *S. enterica* serovar Typhimurium strain 12023 was used as the parental strain for knockout construction and for all other experiments (gifted by Prof. M. Hensel, Germany). It is virulent in the mouse model of infection. The wild type culture was grown at 37°C in Luria broth in nalidixic acid (50 µg/ml), the Δ*argT Salmonella* in kanamycin (50 µg/ml) and complemented Δ*argT* strain in ampicillin (50 µg/ml). Heat killed *Salmonella* was prepared by heating the bacterial culture at 80°C for 20 minutes.

### Preparation of bone marrow-derived macrophages (BMDMs)

As described before [32], femurs were collected aseptically from mice and the marrow was flushed out. The cells were maintained in DMEM supplemented with 30% L929 cell-conditioned medium, 10% heat-inactivated FBS, 2 mM l-glutamine, 100 U/ml penicillin and 100 µg/ml streptomycin. The cells were observed to be >90% CD11b positive by fluorescence-activated cell sorting analysis. The L929 cell line was a kind gift of Prof. M.S.Shaila, Department of Microbiology, Indian Institute of Science, Bangalore, India.

### Cell culture and bacterial infection

Cells were maintained in a 37°C incubator with 5% CO_2_ in Dulbecco's modified Eagle's medium (DMEM, Sigma) supplemented with 10% heat-inactivated fetal calf serum (Sigma). As described before [33] the *Salmonella* strains were added to the macrophage cells growing in 24-well tissue culture plates at a multiplicity of infection (MOI) of 10. Bacteria were centrifuged onto the cells at 500×g for 10 min. After infection for 25 min, the cells were washed thrice with PBS and incubated for 1 h in cell culture medium containing 50 µg/ml gentamicin (Sigma). The medium was replaced with 10 µg/ml gentamicin containing medium for the rest of the experiment. In other set of experiments, the cells were depleted of arginine by culturing in arginine free medium (Hi-media) for 72 h and used for subsequent studies with supplementation of ^14^C- L-arginine (BARC, India, 0.1 mCi/ml).

For the enumeration of the intracellular bacteria, the macrophages were washed three times with PBS and lysed with 0.1% Triton X-100 for 10 min and serial dilutions were plated onto LB agar plates.

### *Mycobacterium bovis* BCG infection

*M. bovis* BCG Pasteur 1173P2 was grown to mid-log phase in Souton's medium. Batch cultures were aliquoted and stored at −70°C. Representative vials were thawed and enumerated for viable colony forming units on Middlebrook 7H10 agar (Difco) supplemented with OADC (oleic acid, albumin, dextrose, catalase). Single-cell suspensions of bacteria were obtained with short pulses of sonication. Bacteria were used at 10 MOI for the infection as described before [34].

### Determination of the nitrite concentration

Nitrite (NO_2_^−^) accumulation in the supernatants of the cultured macrophages was used as an indicator of NO production and was measured by the Griess reaction with sodium nitrite as a standard to calculate the amount of nitrite produced. 50 µl of the supernatant was incubated with 50 µl of the solution containing N-[naphthyl] ethylenediamine dihydrochloride (NED) (0.01%) and 50 µl of the solution containing sulfanilamide (0.1%) in 5% phosphoric acid for 10 min. The absorbance was then measured at 540 nm.

### Semiquantitative RT-PCR

BMDMs were seeded at 1×10^6^/well in six-well plates and infected at 10 MOI with the WT bacteria. After 12 h of infection, the total RNA was isolated using TRIzol reagent (Sigma). Subsequently, 2 µg RNA from each sample was reverse transcribed using ‘PROMEGA RT kit’. One PCR cycle consisted of the following: 94°C for 1 min, 60°C for 1.5 min and 72°C for 2 min. For mCAT1 following primers were used: forward, 5′-caa caa tag gac caa aac acc c-3′ and reverse, 5′-cga aga tgc tca aga cag gaa g-3′. For mCAT2B following primers were used: forward, 5′-tca att cca aaa cga aga cac cag ta**-**3′ and reverse, 5′-agg tca aaa aga aag gcc atc aca-3′. Similarly, for mouse *β-actin*: forward, 5′-tgg aat cct gtg gca tcc a-3′ and reverse, 5′-taa cag tcc gcc tag aag ca-3′ primers were used.

### Arginine uptake assay in BMDMs

Arginine uptake was measured in uninfected BMDMs and in those infected with *Salmonella* at a MOI of 10 as described previously [12]. Briefly, after 12 h of infection, two initial washes were given with 500 µl of prewarmed uptake solution (137 mM NaCl, 5.4 mM KCl, 1.2 mM MgSO_4_.7H_2_O, 2.8 mM CaCl_2_.2H_2_O, 10 mM HEPES and 1 mM KH_2_PO_4_, pH 7.4). Arginine uptake was started by adding 250 µl of 100 µM L-[^14^C (U)] arginine (0.1 mCi/ml, BARC, India) in prewarmed uptake buffer containing 5 mM L-leucine for 10 min in a tissue culture incubator in 10% CO_2_ at 37°C. The reaction was stopped by removing the radioactive arginine and giving three washes with stop solution (10 mM HEPES, 10 mM Tris, 137 mM NaCl and 10 mM non radioactive arginine [pH 7.4]) to remove the unincorporated substrates. Cells were then lysed with 1% sodium dodecyl sulfate and the radioactive incorporation was determined with a liquid scintillation analyzer. The protein concentrations were measured by Bradford reagents. The amount of incorporated arginine per sample was normalized to the total protein concentration of each sample.

### Construction of the *Salmonella* strain expressing the chromosomal ArgT:: 6xHis fusion protein

The *Salmonella* strain expressing the ArgT:: 6xHis fusion protein was engineered in serovar Typhimurium by a modified method from the one-step deletion strategy as described by Datsenko [35]. Briefly, serovar Typhimurium transformants carrying a red helper plasmid (pKD46) were grown in LB with ampicillin and 10 mM L-arabinose at 30°C to an OD (600 nm) of 0.35–0.4 and then made electro competent by washing three times with ice-cold 10% glycerol and MilliQ water. In this strategy, the forward knockout primer was modified to carry a 5′ 6 histidine coding sequences. This histidine tag containing primer was targeted against the region immediately downstream of the *argT* gene (including the *argT* stop codon). The knockout primer set effectively knocked out the 1 kb gene (STM2356) downstream of *argT* while concomitantly tagging *argT* on its C terminal with 6 histidine coding sequences. This was followed by another stop codon so as to obtain only a ArgT:: 6xHis fusion protein.

PCR product containing the chloramphenicol resistance gene (from pKD3 plasmid) flanked by sequences upstream and downstream of the *argT* gene was prepared. following primers were used: forward, 5′caaaaagtacttcgattttaatgtttacggcgatcatcaccatcaccatcactga catatgaatatcctccttag 3′ and reverse, 5′ caaaaagtacttcgattttaatgtttacggcgatcatcaccatcaccatcactga catatgaatatcctccttag 3′. This DNA was then electroporated in *Salmonella* Typhimurium carrying pKD46. The mutants were selected by chloramphenicol resistance and confirmed by PCR using the following confirmatory primers. For confirmation following primers were used: forward, 5′- cctcacatcacgccggat -3′ and reverse, 5′- cgaaggtttcctgaagcag -3′. In the knock in strain, a 1-kb band corresponding to the chloramphenicol cassette was amplified whereas in the WT strain a 1.2-kb band corresponding to the next gene of *argT* gene (STM2356) was observed. We also confirmed the chromosomal knock in strain by lysing the bacteria and then performing an anti His western blot and observed a 27 kDa single band corresponding to the ArgT:: 6xHis fusion protein.

### Expression of the ArgT protein

For this purpose, the *Salmonella* strain expressing the ArgT:: 6xHis fusion protein was used. The wild type *Salmonella* strain was used as a control. Both the strains were inoculated in LB broth and the BMDMs were infected separately with each strain. From the infected cells, bacteria were purified and equal amount of the total protein was loaded in a 15% SDS PAGE. The LB grown bacterial lysate was also loaded in the same gel as a control. The proteins were transferred onto nitrocellulose membrane and anti His western blotting was performed with HRP conjugated anti-His antibody (1∶20000, Sigma). The loading control was Ribosome Recycling Factor (RRF) and anti-RRF antibody (A kind gift of Professor Umesh Vershney, Indian institute of Science, India. polyclonal, 1∶2000) was used for this purpose. We could effectively observe the expression level of the ArgT :: 6x His protein in the infected cells. Further, the change in the ArgT:: 6x His expression was also monitored when the bacteria shifted from LB to intracellular condition.

### Construction of the E. coli :: GFP strain

*E. coli* DH5α strain was made competent by CaCl2 method and the GFP plasmid was transformed by heat shock method. The resultant colonies were selected in ampicillin plates and the presence of the plasmid was confirmed by digestion and the expression of GFP was checked by fluorescence microscopy.

### Construction of the *argT* mutant (Δ *argT) Salmonella* strains

The *argT* (STM 2355) mutation was engineered in serovar Typhimurium following the one-step deletion strategy as described by Datsenko [35]. Briefly, serovar Typhimurium transformants carrying a red helper plasmid (pKD46) were grown in LB with ampicillin and 10 mM L-arabinose at 30°C to an OD (600 nm) of 0.35–0.4 and then made electro competent by washing three times with ice-cold 10% glycerol and MilliQ water. PCR product containing the kanamycin resistance gene (from pKD4 plasmid) flanked by sequences upstream and downstream of the *argT* gene was prepared. For *argT* following primers were used: forward, 5′-acc gtg ata gtt ccc cag cgc ggc gcg tta tcc cct tcc cgt gta ggc tgg agc tgc t-3′ and reverse, 5′-cac aca acg cca cgt aaa aca taa gaa aat gac gcc act tca tat gaa tat cct cct tag-3′. This DNA was then electroporated in *Salmonella* Typhimurium carrying pKD46. The mutants were selected by kanamycin resistance and confirmed by PCR using the following confirmatory primers. For *argT* following primers were used: forward, 5′-ctg ttc cgc aac ggc tta tg-3′ and reverse, 5′-cga atc gtt ttg ctg acg tg-3′. In the knock out strain, a 1.5-kb band corresponding to the kanamycin cassette was amplified whereas in the WT strain a 782 bp band corresponding to the *argT* gene was observed. Another set of primer was used to confirm the knock out strain wherein a kanamycin internal reverse primer and a gene specific forward primer was used. In the knockout strain a 750 bp band was observed and in the WT strain no band was visible. The sequence of the reverse primer was 5′ cagaccgttcagctggat 3′ and the forward primer was 5′-ctg ttc cgc aac ggc tta tg-3′. Further one more set of oligos (which were later used for cloning) was used where the forward primer spans the 5′ and the reverse primer spans the 3′ region of the *argT* gene. The oligos were forward 5′ atgcggatccatgaagaagaccgttctcgc 3′ and reverse 5′ atgcaagctttcaatcgccgtaaacattaa 3′. These primers gave a 750 bp band in the WT strain and no band in the knock out strain.

### Construction of the complemented Δ *argT* (c- Δ *argT*) *Salmonella* strain

DNA extracted from the WT *Salmonella* was used as a template to amplify *argT* gene using forward primer 5′ atgcggatccatgaagaagaccgttctcgc 3′ and reverse primer 5′ atgcaagctttcaatcgccgtaaacattaa 3′. The amplified product was purified and the inserts along with vector pQE60 were digested with BamH1 and HindIII. The vector and insert were mixed at 1∶3 molar concentrations and ligated at 16°C for 16 h. The vector-containing inserts were then transformed into *Escherichia coli* competent cells and plated on LB-carbencillin plates after 1 h incubation in SOC medium. The colonies were screened for plasmid having insert by restriction digestion and the purified plasmid containing *argT* was then transformed into the Δ*argT* electrocompetent cells.

### *In Vivo* Arginine uptake assay

For the determination of the in vivo arginine uptake, 5 days after infection liver and spleen were taken aseptically from either the control or infected mice. The organs were then crushed into single cell suspensions mechanically and dissolved in 1 ml PBS. Each cell suspension was counted and 1×10^6^ cells were taken and plated in 24-well tissue culture plates immediately before use in the experiment. The arginine uptake was measured in a similar manner as described above.

### *In vitro Salmonella* Arginine uptake assay

Overnight grown cultures of the WT and Δ*argT Salmonella* strains were subcultured and grown in LB to stationary phase at 37°C with constant shaking at 115 rpm. The cell density at 600 nm was measured using spectrophotometer and equal OD aliquots of the two strains were taken for the determination of the arginine uptake capacity of each strain. 1×10^8^ bacteria were taken for each sample and washed twice with 500 µl of pre-warmed uptake solution and further processed for the arginine uptake assay as described above. For each sample the amount of incorporated arginine was normalized to the total bacterial protein.

### Estimation of host Arginine incorporation in intracellular *Salmonella*

The BMDMs maintained in the arginine free DMEM were infected with either the WT or Δ*argT* strain. After 25 min of infection, radiolabelled arginine was added to the cells. After 12 h of infection, the intracellular bacteria were isolated from the infected macrophages as described previously [30], [36]. In brief 12 h after infection, cells were lysed on ice by incubating for 30 min in 0.1% SDS, 1% acidic phenol and 19% ethanol in water. *Salmonella* were isolated from the lysate by centrifugation, and total protein was lysed by using bacterial protein lysis solutuion. In each case, bacteria were recovered from a six-well plate of infected cells and pooled to isolate the protein. The bacteria were plated in antibiotic plates to enumerate the number of bacteria present for the different strains. After obtaining the CFU data bacterial number was normalized for the different samples and duplicate wells were used for further experiments and equal amounts of the bacterial proteins after lysing 10^9^ bacteria were loaded onto SDS PAGE. The gel was exposed in the cassette and the incorporated radioactivity in the bacterial lysate was assessed by performing phosphor imager (Fujifilm FLA-5100) scan. Equal amount of the samples were loaded in a different gel and with a positive control of BMDM lysate and after transfer the membrane was probed with anti-RRF antibody and anti-Actin antibody.

### Mice Infection

Six- to eight-week-old BALB/c mice (Central Animal Facility, Indian Institute of Science, Bangalore, India) were maintained under specific-pathogen-free conditions. All procedures with animals were carried out in accordance with institutionally approved protocols. Bacterial strains were grown under shaking conditions overnight at 37°C, centrifuged, washed and resuspended to the appropriate concentration in sterile PBS and administered at 1×10^7^ CFU/mice. For the organ infiltration experiment, 5 days after infection, liver and spleen were taken aseptically. The organs were weighed and homogenized in 1 ml PBS. The homogenate was centrifuged and plated at different dilution to determine the bacterial number.

### Confocal experiments

Infected cells were washed free of medium and fixed for 10 min in paraformaldehyde (3.5%). Latex beads carboxylate modified fluorescent yellow green (Sigma) were added to the cells at a ratio of 25∶1. Fixed cells were then incubated with rabbit anti-mCAT1 antibody (Santacruz) diluted 1∶50 and/or mice anti-mLAMP1 antibody (Dianova) for 1 h in PBS containing 2% BSA, 2% goat serum and 0.2% saponin. This was followed by incubation with goat anti-rabbit IgG conjugated to Cy5 (Jackson's lab, 1∶100) and/or goat anti-mice IgG conjugated to Cy3 (Jackson's lab, 1∶100) for 1 h. Samples were viewed on a confocal laser-scanning microscope equipped with an argon laser (Zeiss, Germany).

### Statistical analysis and software

Each assay was repeated at least 3 times. In vitro data were analyzed by paired t test (two sample, equal variance). Results of mouse *in vivo* challenge studies were evaluated by using Mann-Whitney U tests from the GraphPad Prism 4.0 software. Differences between sets were considered significant for P<0.05. Immunoblots were quantified using Multi Gauge V2.3 software.
